The article "Detection of Aerobics Action Based on Convolutional Neural Network" was published in 2022. Journal: Comput Intell Neurosci.

# Detection of Aerobics Action Based on Convolutional Neural Network

**DOI:** 10.1155/2022/1857406

**Published:** 2022-01-05

**Authors:** Siyu Zhang

**Affiliations:** Sangmyung University Seoul, 20 Hongjimun 2-gil, Jongno-gu, Seoul 03016, Republic of Korea

## Abstract

To further improve the accuracy of aerobics action detection, a method of aerobics action detection based on improving multiscale characteristics is proposed. In this method, based on faster R-CNN and aiming at the problems existing in faster R-CNN, the feature pyramid network (FPN) is used to extract aerobics action image features. So, the low-level semantic information in the images can be extracted, and it can be converted into high-resolution deep-level semantic information. Finally, the target detector is constructed by the above-extracted anchor points so as to realize the detection of aerobics action. The results show that the loss function of the neural network is reduced to 0.2 by using the proposed method, and the accuracy of the proposed method can reach 96.5% compared with other methods, which proves the feasibility of this study.

## 1. Related Work

Object detection, as an important part of the current research field of computer vision technology, mainly detects objects in images or videos. It integrates multiple technologies such as artificial intelligence, and image recognition. So, it is widely used in national defense, military, and other fields [1–5]. Traditional object detection is mainly for simple action scenes. But the scenes in complex environments have been the focus of the current discussion. As a new method of object detection in the current complex scene, the deep neural network can realize feature transformation with its powerful feature extraction ability. It can be seen that object tracking is better achieved.

In previous research, He et al. combined the deep neural network to detect small brown object targets. The results show that small target objects can be accurately detected by the deep neural network, and the accuracy can reach 98.46% [6]. Zheng et al. proposed a multiscale feature fusion method for the problem in the target detection such as occlusion. In this method, a featured channel is constructed based on a directional gradient, and the features obtained by the above feature channels are used as the input of the deep neural network to detect the target [3]. Yan et al. also proposed to use the neural network to simplify and detect the small target objects, but it mainly designed the trunk network of the deep neural network [7]. Feng et al. proposed a multiscale feature extraction method to track targets in optical remote sensing images. The results show that the method can detect images quickly [8]. Based on the above-related research work, this study takes aerobics action detection as the research object. A method of aerobics action detection based on multiscale features is proposed, and it verifies the method.

## 2. Faster R-CNN Model

The faster R-CNN algorithm proposed by Ren Shaoqing is famous for its efficient detection, and other scholars have proposed an improved algorithm based on the faster R-CNN algorithm. The implementation process of the faster R-CNN algorithm is shown in Figure 1 [9, 10].

As can be seen from Figure 1 that, first of all, a convolutional neural network is used to extract the features of the tested image. Then, a network (RPN) is generated by using candidate regions to process the feature maps, and multiple target candidate regions are also identified. Finally, the classification regression network is used to make judgment, and the characteristics within the candidate region are screened; thus, the judgment value is output.

### 2.1. ResNet Deep Feature Network

ResNet-101 network is an important version of the ResNet deep feature network series. It has deep layers and can extract deeper features of the target so as to achieve the effect of effectively expressing the target without causing delay to the network training, network test, and other processes. There is a residual block in the ResNet-101 network [11] shown in Figure 2.

In the residual block shown in Figure 2, the 1 × 1 convolutional layer is able to adjust the number of channels of the feature map, and the 3 × 3 convolutional layer is able to extract feature information. Deep ResNet-101 networks can be established by stacking more residual blocks. The advantage of the ResNet convolutional architecture is that it is able to greatly increase the number of convolutional layers of the neural network to extract the deep semantic information in the image and ultimately accurately express the target to be detected.

ReLU function is used as the activation function by ZF-Net which replaces the traditional sigmoid function and further strengthens the application performance of deep learning neural networks [12–14]. The sigmoid function is able to map the input of continuous variable values into sections 0-1. However, if the input variable value is very small or large, the derivative of the sigmoid function tends to be 0, which makes the gradient disappear during backpropagation, making the network difficult to learn. The ReLU function effectively avoids the above defects, and its mathematical expression is as follows [15]:

(1) $$\begin{array}{c} f\left(x\right)=\max\left(0,x\right). \end{array}$$

### 2.2. Candidate Region Generation Networks

To comprehensively analyze the color, texture, edge, and other information in the image and select the candidate areas for the target to be tested, this process is actually to roughly detect the target test, such can reduce the pressure on the subsequent classification network.

The candidate region generation network selected and used by the faster R-CNN algorithm is a convolutional neural network, shown as follows.

To analyze with the combination of Figure 3, first, the sliding window traverses the feature map by sliding, mapping the features in the pathway at each position into a 256-dimensional feature vector; then, each eigenvector is led into two fully connected layers, exporting 2 × 9 = 18 scores and 4 × 9 = 36 correction parameters, respectively. Each sliding window position contains 9 benchmark rectangular boxes, which are used to correct the benchmark rectangular box after obtaining 36 correction parameters, resulting in 9 candidate regions. In addition, the 18 scores characterize the scoring results of the candidate regions, each corresponding to two scores, representing the probability of containing and not containing targets within the candidate region to be tested.

A benchmark rectangular box was corrected by using four correction parameters *t*_*x*_, *t*_*y*_, *t*_*w*_, *t*_*h*_ to obtain the candidate regions, and the correction formula is listed as

(2) $$\begin{array}{c} x=w_{a}t_{x}+x_{a}, \end{array}$$

(3) $$\begin{array}{c} y=h_{a}t_{y}+y_{a}, \end{array}$$

(4) $$\begin{array}{c} w=w_{a}\exp\left(tw\right), \end{array}$$

(5) $$\begin{array}{c} h=h_{a}\exp\left(th\right). \end{array}$$

In the formula, *x*, *y*, *w*, *h* and *x*_*a*_, *y*_*a*_, *w*_*a*_, *h*_*a*_ represent the center transverse coordinate, center ordinate, width, height of the candidate region, and the benchmark rectangular box, respectively.

Multitask loss function is quoted in the faster R-CNN algorithm, as described as follows [16]:

(6) $$\begin{array}{c} L\left(p,u,t^{u},v\right)=L_{\text{cls}}\left(p,u\right)+\lambda \left[u\geq 1\right]L_{\text{box}}\left(t^{u},v\right). \end{array}$$

In the formula, the classification loss function is as follows:

(7) $$\begin{array}{c} L_{\text{cls}}\left(p,u\right)=-\log\;p_{u}. \end{array}$$

Bound regression loss function is as follows:

(8) $$\begin{array}{c} L_{\text{box}}\left(t^{u},v\right)=\sum_{i\in \left\{x,y,w,h\right\}}\text{smooth}\left(t_{i}^{u}-v_{i}\right),\\ {\text{smooth}}_{Li}\left(x\right)=\left\{\begin{array}{cc} 0.5x^{2}, & \text{if }\left|x<1\right|,\\ \left|x\right|-0.5, & \text{otherwise.} \end{array}\right. \end{array}$$

From the formulas, the purpose of the faster R-CNN training is to minimize the loss function *L*_cls_, minimality of *L*_box_. A target mask is also set to meet the application requirements.

(9) $$\begin{array}{c} t_{x}^{*}=\frac{\left(x^{*}-x_{a}\right)}{w_{a}},\\ t_{y}^{*}=\frac{\left(y^{*}-y_{a}\right)}{h_{a}},\\ t_{w}^{*}=\log\frac{\left(w^{*}\right)}{w_{a}},\\ t_{h}^{*}=\log\frac{\left(h^{*}\right)}{h_{a}}. \end{array}$$

In the formula, *x*^*∗*^, *y*^*∗*^, *w*^*∗*^, *h*^*∗*^ represent the center abscissa, center ordinate, width, and height of the target label box.

### 2.3. Principle of the Pooling of the Spatial Pyramid

Space pyramid pooling (SPP) can map local features and fuse the space of different dimensions with the advantage of the ability to generate fixed-size feature vectors and improve the adaptability of the convolutional neural network structure. The working principle of the SPP is shown in Figure 4.

To analyze with Figure 4, SPP contains multiple scales of pooling layers that can be applicable to convolutional layer features of any size and finally output eigenvectors of fixed dimensions.

## 3. Method Improvement

The faster R-CNN algorithm remains to be improved when handling multiscale problems, for which this paper introduces the feature pyramid network (FPN) into the faster R-CNN framework. The improved algorithmic framework is shown as below in Figure 5.

Combined with the analysis in Figure 5, the original image is feature extracted by using ResNet. Considering the several layers in ResNet output feature maps of the same size, the comparative analysis found that the feature map of Conv1 occupies too much memory. So, only the output of Conv2∼Conv5 after nonlinear activation is used as the reference feature map for the current stage; then, Conv2–Conv5 are obtained [17].

The positive and negative labels of the anchor are set based on the current anchor intersection ratio (IOU) to the actual position of the target to train the RPN network. The modified RPN network slides a network head at all levels of the FPN network to determine the regional location that may contain the target to be tested, and the improved RPN network maintains a high level of parameter sharing.

The improved low-level feature map of the FPN feature pyramid has high-resolution characteristics, can extract deep semantic information, and can achieve accurate retrieval of multiscale and small goals.

### 3.1. FPN Multiscale Features

The FPN network has an advantage in multiscale target detection to introduce it into the faster R-CNN that can further improve the model adaptability to multiscale target, small target detection based on maintaining the efficiency of model detection. The FPN network is able to accept pictures of any size, configure them in the CNN convolutional neural architecture, and can more effectively extract deep feature maps. According to the requirements of each convolutional layer of CNN, the feature graph corresponding to the proportional size is then output respectively, thus establishing the feature graph pyramid. It is shown here that the FPN network is able to output feature maps of different scales and also to integrate feature maps at different layers. The realization process of this function is that the FPN network first sorts the feature maps of all layers in the CNN network, then magnifies the length and width of the deeper feature maps to 2 times of the original, and adds to the feature maps of the corresponding shallow layer, thus realizing the fusion operation between the feature maps at different levels. After this operation, the shallow feature map contains both deep semantic information and a high-resolution ratio, thus improving the detection accuracy for multiscale targets.

### 3.2. The Multiscale Multiplayer Aerobics Action Target Detection Algorithm of CNN

After above optimized processing, the finally established multiscale RPN can accurately extract multiscale ROIs as well as multiscale human targets.

#### 3.2.1. ROIs Extracted from Multiscale RPN

Using the FPN for the RPN stage is able to extract multiscale candidate regional ROIs. In different layers of the FPN, ROIs were extracted from sliding anchor point, and the score and regression position of each candidate region were determined. Although the improved RPN stage contains multilayer feature maps, there is no need to extract ROIs independently. Instead, pooling the anchors is acquired by the layers within the same set, from which higher scoring regions were selected as ROIs. The loss function cited in this process refers to [18]

(10) $$\begin{array}{c} L_{1}\left(\left\{p_{i}\right\},\left\{t_{i}\right\}\right)=\frac{1}{N_{\text{cls}}}\sum_{i}L_{\text{cls }I}\left(p_{i},p_{i}^{*}\right)+\lambda \frac{1}{N_{\text{reg}}}\sum_{i}p_{i}^{*}L_{\text{reg }1}\left(t_{i},t_{i}^{*}\right). \end{array}$$

In the formula, *i* refers to the serial number of anchors in a small training batch, *L*_1_ refers to the total loss function of the RPN stage, *p*_*i*_ is the probability of predicting the *i* anchor as the target, *t*_*i*_ is the RPN stage prediction, *t*_*i*_^*∗*^ is the real boundary box position of the target, using *p*_*i*_^*∗*^ to discriminate positive and negative anchors, *N*_cls_ indicating the size of a small batch of training, *N*_reg_ is the number of anchors, *λ* as the balance parameter, and *L*_reg 1_ is the regression loss function which uses the smooth *L*_1_ loss.

Considering that the feature maps at each layer of the FPN have different scales, this subsection uses only a single-scale anchor, such can enable the improvement of the multiscale target detection effect.

Using the IOU as the classification basis, the anchors contain two categories as positive and negative anchors. However, if there are only small-scale targets in the image and the number of small-scale targets is small, the ratio of negative and positive anchors obtained based on the RPN network is too large, which means that the extracted background semantic information is too rich but affects the feature extraction effect on the foreground target, and the obtained target detector for the foreground target identification effect is not ideal. To avoid this problem, it is necessary to reasonably limit the number ratio of positive and negative anchors generated in the RPN stage to prevent interference with the target detection effect due to the too large ratio.

This paper studies the problem of aerobics action object detection. Combined with the morphological characteristics of the aerobics action, the anchor aspect ratio is set at 1 : 2, 1 : 2, 1 : 1, 2 : 1, and 1 : 3 in the paper, which can maintain the detection efficiency and detection effect of the neural network for the aerobics action target.

#### 3.2.2. Multiscale Aerobics Action Target Detector

The aerobics action target detection network uses the FPN feature pyramid to extract the characteristics of the aerobics action target. The realization process is according to the scale of the ROls output by RPN, corresponding to the corresponding layer of the feature pyramid, and it then extracts the target features. Deep feature maps have been extracted at the FPN stage, where it is only necessary to extract fixed-size target feature maps using ROI pooling and then input the extracted features into the fast R-CNN target detector. The target detector has 2 full connection layers in the front to assess the confidence of the target while performing a regression analysis of the target region. The loss function of this procedure is listed in the below equation [19, 20]:

(11) $$\begin{array}{c} L_{2}\left(p,u,t^{n},v\right)=L_{ds2}\left(p,u\right)+\delta \left[u\geq 1\right]L_{\text{loc}2}\left(t^{M},v\right). \end{array}$$

In the formula, *L*_2_ represents the total loss function of the second stage target detection, *L*_cls2_ represents the classification loss, *L*_loc2_ represents the smooth *L*_1_ regression loss function, [*u* ≥ 1] represents the rank indicator function, *u* represents the true category of the target, *p* represents the confidence level of the predicted target, *t*^*n*^ and *v* represent the prediction boundary box corresponding to the *u* category and the position of the real boundary box respectively, and *δ* represents the equilibrium parameter.

Previous studies are conducted on whether target detectors at the fast R-CNN stage share parameters at different FPN layers, confirming that the differences between different layers were small. Thus, this paper decides to share the weights between different layers of the feature pyramid hierarchy, such can effectively improve the target detection efficiency.

## 4. Experimental Analysis

### 4.1. Experimental Environment and Dataset

This experiment uses the Ubuntu 16.04 version of the Linux system, and the server configuration conditions are Intel@Xeon@CPUE5-2678v3@2.50 GHz, NVIDIA GeForceGTX 1080 Ti, and 32 GB of memory. The deep learning framework used in this experiment is that TensorFlow-GPU 1.10, which is equipped with cuDNN 6.0, CUDA 8.0 and has an Anaconda3 version of the Python library as well as Python 3.5.

To meet the needs of target detection of aerobics movements, the aerobics action of this experiment was equipped mainly acquired through the collection.

### 4.2. Training Results and Analysis

This experiment selects the faster R-CNN model and uses the feature map of various FPN layers to detect the human targets, in order to achieve the multiscale target detection effect. To achieve the goal, the number ratio of positive and negative anchors in the RPN is limited in this experiment to prevent interference with the human object detection effect due to the too large ratio. Combined with the morphological characteristics of the human body, the anchor aspect ratio was adjusted, and a 3 : 1 proportional scale was added, which can more accurately identify the human targets. After this improvement, coordinating with INRIA, PETS 2009, and Caltech, three standard datasets, the aerobics action target can be detected effectively.

Taking the above dataset as an example, the TensorBoard tool is used to demonstrate the training process of neural networks, specifically as follows:

First, the visualization results of the feature maps of each layer of the FPN network are shown in Figure 6.

Figure 7(a) shows the feature map output of layers 2–5 of the feature extraction network, with the layer map of C2–C5 from bottom to top; Figure 7(b) shows the feature map output of layers 2–5 obtained after the introduction of FPN and layers P2–P5 from bottom to top. In comparison, although the semantic information contained in the C5 layer and P5 layer feature maps is basically similar, there is a large gap between the semantic information contained in the C2 layer and P2 layer feature maps.

Raw images were input into the RPN network, and the RPN network detected the candidate region ROIs and to score each candidate region ROIs. After the introduction of the FPN pyramid architecture, four-scale feature maps are output at the RPN stage, corresponding to four layers, and the number of ROIs output from each layer is shown in Figure 7.

In Figure 7, the number of ROIs in P2∼P5 layers of FPN is shown, respectively, in which the number of ROIs in lower-level feature maps is significantly greater than the number of ROIs in high-level feature maps. The cause is that the Caltech dataset used for training contains a large number of small-scale targets, while the number of large-scale targets is significantly less, which interferes with human target detection.

Variation tendency in the values of various loss functions in the improved RPN stage is shown in Figure 8.

For the analysis combined with Figure 8, the value of the RPN loss function fluctuates as the number of training iterations increases, but the overall trend remains to decrease, and the total loss value of the RPN stage decreases from 0.12 to 0.02. Thus, it is seen that the trained ROIs regions suggest that the network can accurately extract human target candidate region to enter higher-rated ROIs into the second stage fast R-CNN target detection framework, then output two-loss values, namely, boundary box regression loss and classified loss, with trends shown in Figure 9.

For the analysis combined with Figure 9, with the number of training iterations increases, all three curves show some volatility, but the overall trend decreases, and the total loss value in the fast R-CNN phase decreases from 0.9 to 0.2. It can be seen that the ability of the target detection network to detect human targets is gradually fitted to the datasets used for training.

The trend of overall loss function values of the entire neural network is outlined from the trial data, as shown in Figure 10.

Combined with Figure 11, as the number of iterative training increases, the overall loss value of the whole neural network decreases from 1.7 to 0.8, which indicates that the trained neural network can more accurately detect aerobics movement targets.

To circumvent overfitting during training, this experiment limited the weight attenuation, that is, to maintain a negative correlation with the update weights of the neural network and the number of training iterations during training, under which the trend of update weights is shown in Figure 11 below:

Combined with Figure 11, with the increasing of number of training iterations, the updated weight decreases from 0.627 to 0.581.

### 4.3. Comparison of Experimental Results

The baseline faster R-CNN is compared. Meanwhile, average accuracy was used as the algorithm performance (AP) evaluation index, with an AP value equal to the lower area of the PR curve. From the perspective of the application effect, by combining the precision-recall diaries under different threshold conditions, the comprehensive index AP of the target detection accuracy is obtained, which can objectively and comprehensively evaluate the algorithm detection accuracy. The average accuracy AP values of the baseline faster R-CNN, CNN, R-CNN, and Mask R-CNN, the method in this paper summarized in Figure 12.

According to Figure 12, the average accuracy AP value of the baseline faster R-CNN is 90.7%, the average accuracy AP value of the proposed algorithm is 96.5%, 91.1%, and 88.6%. By comparison, the method of this paper is based on faster R-CNN. Object features were extracted by using FPN, combined with the correlation optimization algorithm to achieve a higher ground detection accuracy generally and significantly outperformed the detection accuracy of the baseline faster R-CNN model.

## 5. Conclusion

In summary, it is difficult to adapt to the detection needs of multiscale and small target application scenarios in the process of aerobics action target detection. Therefore, this paper proposes a multiscale and multitarget aerobics action target detection algorithm based on CNN network architecture. After introducing the two-stage target detection framework of the faster R-CNN model, this paper systematically analyzes the process of using the ResNet deep main network to extract and utilize the process of multiscale target feature extraction by using the FPN network. Then, the FPN feature pyramid was fused separately in the two stages of the faster R-CNN framework to construct a multiscale RPN proposal network as well as a multiscale aerobics action objective detector to set the number of positive and negative anchors reasonably is conducive to improving the detection efficiency of the aerobics action targets of the algorithm. Limiting the vertical and horizontal ratio of anchors scientifically and also optimizing the overall neural network can improve the detection effect of multiscale and multiperson aerobics movements. Finally, in this paper, baseline faster R-CNN methods were used for comparison experiments separately. Finally, confirming the baseline faster R-CNN, this method in the paper can achieve preferable detection results. The innovation of this study is to identify the aerobics movement from the perspective of target detection and recognition so as to provide more reference paths for the auxiliary training of sports.

## Figures and Tables

**Figure 1:** Faster R-CNN structure.

**Figure 2:** A residual block of the ResNet-101.

**Figure 3:** The candidate region generation networks.

**Figure 4:** Principle of spatial pyramid pooling.

**Figure 5:** Basic framework of improved fast R-CNN.

**Figure 6:** Comparison of the feature maps at each level of the FPN network. (a) Original feature map. (b) FPN feature map.

**Figure 7:** The number P2∼P5 of ROIs from multifeature graph. (a) P2. (b) P3. (c) P4. (d) P5.

**Figure 8:** Loss function value in the RPN stage.

**Figure 9:** Loss function value in the second stage detection. (a) Classified losses in the second stage. (b) Returned losses in the second stage. (c) Total losses in the second stage.

**Figure 10:** Loss function value of total neural network.

**Figure 11:** Neural network weight attenuation.

**Figure 12:** Baseline fast R-CNN and proposed method.

## Data Availability

The data are available from the corresponding author upon request.
